# Evaluation of College English Teaching Quality Based on Improved BT-SVM Algorithm

This article has been retracted.

**DOI:** 10.1155/2022/2974813

**Published:** 2022-08-19

**Authors:** Minsheng Lou

**Affiliations:** Jinhua Advanced Research Institute, Jinhua 321000, China

## Abstract

With the development of teaching evaluation program, colleges and universities have reformed according to the actual situation of the school. With the development of evaluation activities, many universities are eager to establish their own teaching quality evaluation system, so as to pre-evaluate the teaching quality of schools. SVM is one of the most widely used machine learning algorithms that enables efficient statistical learning with a very limited number of samples. Considering the excellent learning performance of SVM, it is very suitable for the teaching quality evaluation system. In this paper, we optimize the existing multiple classification algorithm for binary trees and propose a new method. Learning the popular teaching quality evaluation system in colleges and universities, the binary tree support vector machine classification algorithm, and design comparison experiment, the experimental results show that the evaluation model proposed in this paper has strong generalization ability and higher classification accuracy and better classification efficiency.

## 1. Introduction

In order to improve the cultural quality and meet the demand of rapid economic development for new talents, China has carried on the major reform of higher education system, many university enrollment scale for four consecutive years, which means that the end of the era of higher education “elite education” began to enter the “popular education” [1]. As one of the three major subjects, English teaching is the same as every previous reform, with both advantages and disadvantages [2]. After some universities, due to the influence of many factors (such as the lack of teaching resources, teachers, the quality of students, etc.), the quality of English education in schools has shown a downward trend [3]. University administrators are trying to improve the quality of English teaching, but to ensure success without additional manpower and material resources. Teachers are the implementers of school teaching activities, and they play an irreplaceable core position in the teaching work [4].

There is a direct relationship between the teaching quality of college English and the teaching mode of teachers [5]. Generally speaking, when a school has stronger teachers, it can win the favor of students and parents in local areas and even other regions. From the perspective of the government, more resources will be invested in the school to further enhance the influence of colleges and universities and cultivate more high-quality talents for the society [6]. It can be seen that it is an inevitable trend of future education to enhance students' knowledge level by improving the teaching quality of teachers. Colleges and universities design high-quality learning activities according to students' actual learning situation and data combing, combined with teachers' teaching experience, so as to build an effective teaching mode for students [7].

The current academic research focus on the evaluation of teaching quality in colleges and universities. With the deepening of informatization, domestic and foreign colleges and universities and teaching quality evaluation are more and more valued by colleges and universities. Through the evaluation of teachers' teaching quality, it is found that teachers' teaching mode and activity deviation are effective suggestions for improvement, providing favorable conditions for improving the quality of teaching [8]. At present, Internet technology has been related to many industries, and the evaluation method of English teaching in universities in the information age has changed the original teaching evaluation mode [9]. However, in China, whether for teaching evaluation, especially English teaching evaluation, the practice of research and practices are relatively short, which requires scholars and education departments to pay more attention to teaching evaluation and formulate a scientific and reasonable evaluation system of English teaching quality in universities.

## 2. Related Research Results

### 2.1. Research on Teaching Quality

The research on teaching quality evaluation abroad started relatively early, the first student questionnaire appeared in 1915, and so far, Western scholars on teaching quality evaluation have a history of nearly a hundred years. In the early twentieth century, many European and American countries began to explore the establishment of teaching evaluation system, but only a few schools had formal evaluation procedures for fair and effective evaluation of teacher teaching, not established until the 1950s [10–14]. After a hundred years of development, every Western university generally has a relatively complete evaluation system, and the evaluation activities are very stable, but our education system is very different from that of Western countries. Therefore, domestic universities should, according to their own characteristics, and combined with the background of the times, to find the evaluation mode and evaluation method suitable for our school.

In China, the research of education evaluation activities started late. The earliest activity to evaluate teachers ‘teaching quality in Chinese universities occurred in 1984 (held by Beijing Normal University, which aims to provide a reference for measuring teachers' teaching situation). The first clear evaluation of education was in May 1985, when the state promulgated the Decision of the CPC Central Committee on Education System Reform; in June 1985, the first national education evaluation seminar, namely, the Special Seminar on Higher Engineering Education Evaluation, was held in Heilongjiang. At the present stage, the teaching evaluation of teachers in Chinese colleges and universities has entered the stage of in-depth development. The biggest progress in this stage is that colleges and universities pay more and more attention to the student-oriented education concept. School administrators often use students' evaluation results as a reference for teachers' personnel decisions. Most importantly, the teachers, according to the students' feedback, carefully analyze the advantages and disadvantages in the teaching process, and change the teaching methods in time to achieve the purpose of improving the teaching quality.

### 2.2. Research on Multiple Classification Algorithms for SVM

SVM was originally proposed for the double classification problem and cannot be directly used to solve the multi-classification problem. After deeply learning the basic theory of SVM, the researchers have proposed many feasible methods to transform the traditional SVM for multi-classification problems. At present, there are two most commonly used solutions: one is the direct method, which regards the original multi-classification problem as a planning problem, and then optimizes the problem as a whole. The other is the indirect method, which is solved by splitting the multi-classification problem into multiple dichotomy sub-problems [15]. Due to the large calculation amount and long time consuming, direct method is rarely used in practical application, but indirect method is more and more favored by researchers. Scholars propose the all-and-one algorithm that combines one-to-many and one-to-one methods to solve the multi-classification problem [16–19]. A and O. briefly propose the species-directed acyclic graph support vector machine, which uses the idea of directed acyclic graph to combine binary classifiers in one-to-one methods to reduce the test time [20]. Scholars propose the error correction coding support vector machine, which applies the error correction algorithm to multiple classification. Scholars propose the half-against-half method, which uses hierarchical clustering when training a classifier to equally divide the training samples into two subsets that are disjoint. On the basis of combining the advantages of binary tree structure, a multiclassification algorithm is proposed [21–27].

To sum up, the advantages and disadvantages of teaching quality evaluation at home and abroad analyze the advantages and disadvantages of the existing SVM multi-classification algorithm, and the concept of relative distance is introduced into the SVM multi-classification algorithm as the standard to measure the degree of difference between the two categories. In the process of forming a binary tree structure, some snow disasters follow the principle of the easiest separation, first segmentation, minimizing the error, and the accuracy of the accumulation of classification results. There are many existing binary tree support vector machine classification algorithms, and the entire algorithm process is described to verify the results of the study by means of experiments.

## 3. Construction of College English Teaching Quality Evaluation Model Based on Improving BT-SVM Algorithm

### 3.1. Improved BT-SVM Algorithm

Although the binary tree method has many advantages, a new problem appears: how to make the structure of the binary classification tree tend to be a more ideal state. The structure of the binary tree is directly related to the performance of the algorithm, and the SVM binary classifier closer to the root junction has a greater impact on the classification results. Therefore, for those categories that are easier to separate, they should be segmented at small hierarchical knots, so that the constructed optimal super-plane obtains better classification performance.

In practice, as the information available is very limited, therefore, training samples are commonly used to estimate the ease between categories. The usual practice is to express the Euclidean similarity by the Euclidean distance between categories. Although the method is simple, it is only feasible with small overlap between classes. When the overlap between them is large, interclass distances can no longer completely truly reflect the variability of the two classes. For this problem, this paper uses the relative distance between the classes to measure the degree of difference between the two classes. The distance of centers and the distribution of samples are also considered. In comparison, more scientific and feasible laws are defined as follows: let *X* be a sample set of *k* categories, X_i_. For the training set of class *i*, the sample center of class *i* is

(1) $$\begin{array}{c} c_{i}=\frac{1}{n}\sum_{x\in X_{i}}x, \end{array}$$

like *c*_i_, *c*_j_. For the sample centers of classes *i* and *j*, respectively, the Euclidean distance between classes *i* and *j* is

(2) $$\begin{array}{c} d_{ij}=\|c_{i}-c_{j}\|. \end{array}$$

Minimum supersphere radius of class *i* is

(3) $$\begin{array}{c} R_{i}=\max\left\{{\|c}_{i}-x_{i}\|\right\}, \end{array}$$

among *x*_i_ samples for class *i*.

Define 3.4 if the minimum supersphere radius of classes *i* and *j* is *R*_i_ and *R*_j_, respectively, and the Euclidean distance between them is d_ij_, then the relative distance between class *i* and class *j* is

(4) $$\begin{array}{c} D_{ij}=\frac{d_{ij}}{R_{I}+R_{J}}. \end{array}$$

According to the above formula, the relative distance contains two indicators: the Euclidean distance between classes and the minimum supersphere radius. As mentioned above, the Euclidean distance of the two class centers indicates the separation of the samples between the two classes in space, the larger the Euclidean distance between the two classes, the farther apart the two classes are, and the more likely to be separated, while the minimum hypersphere radius reflects the size of the distribution range of the sample in space. The relative distance can simultaneously reflect the distance between two classes and the intersection of sample distribution, that is, Di; the larger the separation of classes *i* and *j*, the better the easier to divide; otherwise, there is less separation between them. The two classes shown in Figure 1, with the one on the left, have higher separability than the one on the right due to the different sample distributions.

### 3.2. Structure of Incomplete Binary Trees Based on Relative Distances

For the binary tree multi-classification SVM, the structure of the binary tree has a very large impact on the performance of the classification system, such as partial and complete binary trees, whose classification performance is different. In the classification problem, training time and classification accuracy are two important indicators to measure the performance of the classification system. Although the number of subclassifiers is the same, in the training stage, most of the subclassifiers in the partial binary tree structure contain relatively many samples, so its total training time is more than the complete binary tree structure. Scholars have proved through experiments that the SVM algorithm of complete binary tree structure has the most ideal classification effect, but in practical classification problems, it is difficult to generate a complete binary tree structure for each problem. For this problem, this paper proposes an incomplete BT-SVM method based on relative distance.

In the incomplete binary tree classification based on relative distance, combining the basic idea of clustering, the two classes with the largest relative distance are determined first, and then the positive and negative classes of the binary classifier are determined according to the distance between the two classes. The whole algorithm follows the principle of the most separable class first segmentation. Here is an example to illustrate the algorithm as the process of constructing a binary tree structure: let the relative distance matrix *D* of the five categories be

(5) $$\begin{array}{c} D=\left[\begin{array}{c} \begin{array}{ccc} 1 & 2 & 10\\ 1 & 3 & 1\\ 1 & 4 & 8\\ 1 & 5 & 4\\ 2 & 3 & 5\\ 2 & 4\; & 2 \end{array}\\ \vdots \end{array}\right]. \end{array}$$

### 3.3. Arithmetic Statement

Incomplete BT-SVM multi-classification algorithm is divided into two parts: training stage and test stage, which are described as follows:

#### 3.3.1. Training Phase

(1) For the preprocessing of the training sample dataset, the first is the normalization processing, and then the standard marks of all categories are stored in the set *C* from small to large.
(2) For classification problems including *k* categories, the relative distance matrix *D* between classes *i*, *i* (*i* = *j*) is calculated according to the formula given above:
  (6) $$\begin{array}{c} D\left[\begin{array}{ccc} 1\;\; & 2 & D_{12}\\ 1\;\; & 3 & D_{13}\\ \cdots & \cdots & \cdots \\ k-1 & k & D_{k\left(k-1\right)} \end{array}\right]. \end{array}$$

#### 3.3.2. Testing Stage

The decision function *D* calculates the 1(*x*) value of the unknown sample x at the root node of the binary tree. If *D*_1_ for(*x*) > 0, the left subtree enters the root node, and the value of the decision function *D*_2_(*x*) is calculated. If it is still greater than 0, continue to enter its left subtree is judged, otherwise it enters its right subtree; if *D*_1_(*x*) < 0, then go to the right subtree of the root node, calculate the *D*_2_(*x*) value, if it is greater than 0, enter the left subtree to judge, otherwise, enter right subtree, loop until the node, and output the class label of the unknown sample, that is, the class label stored in the leaf node.

For binary tree methods, the number of SVM classifiers to be constructed is k-1 regardless of their structure, but the number of training samples for each classifier is not necessarily the same. In the complete binary tree method, the 2nd layer has ii -1, the number of training samples in each layer is the total number of samples. Assuming that the number of classifier samples on the same layer is the same, the training time of this method is

(7) $$\begin{array}{c} T=c\sum_{i=1}^{h}\left(2^{i-1}{\left(\frac{n}{x^{i-1}}\right)}^{2}\right)=cn^{2}\left(1+\frac{1}{2}+\cdots +\frac{1}{2^{h-1}}\right)\approx 2cn^{2}. \end{array}$$

From the above analysis and comparison, we know that when *k* is relatively large, the time cost of incomplete BT-complete multi-classification algorithm of SVM in the training stage is less than that of O V R method, but also greater than O V O method. In the test stage, the time cost is also the smallest, because the test samples need to pass through the least number of classifiers, up to k-1.

### 3.4. Construct the Evaluation Index System of College English Teaching Quality

In my country, with the requirements of the new curriculum reform on teaching quality, effective teaching activities should be made according to the teaching environment of colleges and universities, which also puts forward higher requirements for English teachers, not only need to master a wealth of English knowledge but also according to the individual characteristics of students' teaching environment. Based on the support vector machine evaluation model, the evaluation mode of English teachers' teaching quality is formulated, is classified according to different evaluation results, and effectively uses the evaluation results to improve the work efficiency of English teachers, which is also an inevitable trend for English teachers to teach in the Internet era.

In order to understand the data of English teaching in universities in more detail, the research results and information of evaluation indicators related to English primary schools are collected and sorted out, and the evaluation index setting of this paper is sorted out. The specific content is listed below.

The evaluation index in Table 1 has 4 first-level indicators and 14 second-level indicators, and the value of each second-level index is 100 points. This kind of evaluation table is very common in Chinese universities. It extracts the general common requirement characteristics of all these courses from different types of courses as the evaluation indicators, so it is applicable to the courses of different subjects and different grades. The advantages of this teaching evaluation index are as follows: first, its form is very simple and makes people clear at a glance, and the evaluator is easy to understand and make a judgment. Secondly, the same index system is used to investigate the overall teaching situation of different English teachers, so that school administrators can guide and grasp the realization of teachers' teaching objectives. The implementation process is simple, and the evaluation results are strong.

### 3.5. Construct the BT-SVM English Teaching Quality Evaluation Model

Based on the research of English teaching quality evaluation in the above research, the evaluation system of teaching quality is proposed by finding the problems existing in the teaching evaluation process. By combing the previous research results, the BT-SVM teaching quality evaluation model is used to evaluate the English teaching quality in universities, which makes the effective use of the evaluation results to improve the effectiveness of the teaching evaluation.  Figure 2 shows the teaching quality evaluation model of this paper.

In order to explain the information of the evaluation model, the multi-evaluation module and classification module are explained. First of all, the evaluation module is the process of processing the data after collecting and sorting out the specific information of the evaluated object. Secondly, the classification module is a process of comprehensively evaluating the quality of teachers' English teaching after data analysis, and finally combining them with decision functions. The reason why SVM model is used for analysis is also because it combines information technology to improve the accuracy and computational efficiency of multi-classification algorithm. On the other hand, the SVM model can integrate the campus network, and the whole evaluation process of teachers can analyze the data after sorting out various types of resources to understand the specific situation of the evaluation objects.

## 4. College English Teaching Experiment Based on Improved BT-SVM Algorithm

This experiment takes the dataset in the project “Research and Practice of Quality Assurance of English Teaching Process in College and Quality Evaluation System of English Teaching.” The project is organized by the teaching reform of universities. The operation process of the experiment is shown in Figure 3.

### 4.1. Data Preprocessing

The dataset for this experiment has 337 sample data, of which 287 are training data sample sets, and the remaining 50 serve as test sample sets. Each sample contains 14 feature attributes; that is, a feature attribute corresponds to an evaluation factor in the evaluation index system, and the value range of each attribute is [0, 100]. The teaching quality evaluation model proposed in this paper automatically divides teachers into excellent and poor according to the average score of English teachers. The final output indicates excellent grade, 0 indicates good grade, and 1 means poor grade.

Since the attribute value of the sample is in the range of 0–100, in order to ensure the centralization of the sample data and the effectiveness of the evaluation results, the sample data must be normalized to the sample data 48 times before training the sample. By observing the sample data, it is found that the attribute values of most samples are concentrated within [70, 100], so this paper uniformly normalized the sample data according to the expression (x80)/80 to reduce the time consumption of the training process. The normalized sample data are shown in Figure 4.

### 4.2. Build a Relative Distance-Based BT-SVM Classifier

The modified algorithm is used to train the training sample data to construct a SVM multi-classification model based on the incomplete binary tree structure. This process can be completed in two steps: the first step is to construct the incomplete binary tree structure based on relative distance, and the second step is to train an optimal hyperplane in the method of each leaf node of each incomplete binary tree to obtain an incomplete binary tree support vector machine classifier. The specific operation process is as follows:

The relative distance matrix *D* of the three categories in the training sample dataset is calculated according to the above formula:

(8) $$\begin{array}{c} D=\left[\begin{array}{ccc} 1 & 2 & 0.0531\\ 1 & 3 & 0.0786\\ 2 & 3 & 0.0351 \end{array}\right]. \end{array}$$

Incomplete two-tree structure.

In dataset *C* = {1, 2, 3}, the two categories with the largest relative distance in array *D* were found 1,3 and deposited to dataset C in size order_1_, C_2_. In, i.e., *C*_1_ = {1}, *C*_2_ = {3}. For the remaining category 2, the relative distance between it and category 1, 3 was first found in *D*, and then the size of these two relative distances was compared and added to C if the relative distance between it and category 1 is small_1_In and otherwise placed in C_2_ owing to *D*_12_ > *D*_23_. Therefore, the category label 2 is added to the C_1_In, making the *C* = {1,2}. The following binary trees are constructed with C as the root node, and C1 and C2 as the left and right nodes, respectively:



Then, continue to construct the binary tree with the left subtree as the root node, and finally get the following binary tree structure:



Construct the decision function at each nonleaf node of the binary tree.

For the first time, the 1 and 2 samples are positive in the second time, in the 1 sample and 2 sample, the construction of support vector machine multi-classifier based on relative distance is completed. The trained incomplete binary tree support vector machine multi-classifier was saved to the model file for test phase calls.

### 4.3. Test Performed on the Test Dataset

Open the model file and call the incomplete binary tree support vector machine multiple classifier to test the test sample set. All the test sample data are input to the root junction, and its decision function *D* is calculated_1_(*x*) value; if the *D*_1_(*x*) < 0, then the data belong to category 3, output 3, if *D*_1_. For (*x*) > 0, the decision function *D* is used_2_(*x*). Continue with the judgment; if the *D*_2_(*x*) > 0, the data belong to category 1 and output 1; otherwise, it belongs to category 2 and output 2.

### 4.4. Experimental Results and Analysis

In this experiment, partial BT-SVM multi-classification algorithm is selected as the reference. Partial binary tree divides a category at will at each time during training, which is simple and easy to implement. It is one of the most widely used multi-classification methods in the classification field, and it is selected as the reference to be more comparable. Because the partial BT-SVM algorithm randomly determines which classes are the first to be separated, with high randomness, the fluctuation of classification accuracy may be relatively large; that is, the stability of the algorithm is poor. To prove this statement, this paper uses the partial BT-SVM algorithm and the improved BT-SVM algorithm. Figure 4 shows the accuracy of the partial BT-SVM algorithm in 7 experiments, while the improved algorithm is all 98.93% accurate.

According to the experimental results, we can see that the classification accuracy with the partial BT-SVM algorithm was different, up to 98.20%, and the lowest to 95.69%. The difference is 2.51%, and the fluctuation range is relatively large. This shows that partial BT-SVM algorithm cannot guarantee the accuracy of classification; namely, the algorithm is unstable; when the classification dataset contains categories and data comparison, classification accuracy will be more unstable, because with the increase of categories, each subclassifier chooses the combination of positive and negative class which also becomes more; this is bound to increase the instability of the algorithm. For the modified BT-SVM algorithm, the results of the experiment tend to stabilize in the same experimental environment because the structure of the binary tree is determined.

The time consumption and classification accuracy of the two algorithms are calculated in Table 2, and the values are the mean of the data from seven experiments.

It can be seen from Table 2 that the classification time of the two algorithms is almost the same, mainly because the categories and quantities of experimental data are small, and the amount of calculation is small, so that the classification time of the two algorithms is not obvious. However, As the experimental data categories increase, the depth of the partial BT-SVM algorithm tree increases faster, and the time gap between the two algorithms becomes larger and larger. Moreover, because the improved algorithm uses the relative distance between categories as the criterion to judge which categories should be segmented first, it reduces the error accumulation phenomenon induced by the binary tree structure, so its classification accuracy is relatively high. Therefore, it is feasible to apply the relative distance-based incomplete BT-SVM multi-classification algorithm proposed in this paper to the university English teaching quality evaluation system.

## 5. Conclusion

This paper first provides an overview of the research status of multiple classification algorithms based on SVM, the evaluation of the teaching quality of college English teachers, and its related basic theories. After studying the existing SVM multi-classification methods, we propose an incomplete BT-SVM multi-classification algorithm that measures the phase specificity of classes using the relative distance between classes. This paper designs a prototype framework for English teaching quality evaluation based on improved algorithms. And the experimental results show that the incomplete BT-SVM multiple classification algorithm can effectively improve the accuracy of the classification results.

In general, the main work of this paper is as follows: after deeply analyzing the shortcomings of the existing SVM multi-classification algorithm, this paper puts forward an incomplete BT-SVM multi-classification algorithm. Unlike other distance algorithms, the Euclidean distance of the class center to measure the difference between the categories considers the influence of the class center distance and sample data distribution on the last classification results. The experimental results show that the algorithm can more effectively evaluate the quality of college English teaching.

## Figures and Tables

**Figure 1:** Comparison of two categories at equal distances.

**Figure 2:** Basic incomplete binary tree SVM teaching quality evaluation model.

**Figure 3:** Operation process of English teaching evaluation.

**Figure 4:** Classification accuracy of 7 random experiments with the partial BT-SVM grate method.

**Table 1:** Evaluation indexes of teaching quality of college English teachers.

First-level evaluation indicators	Secondary evaluation index
Content of courses	1. Teaching objectives are clear, the teaching content meets the requirements of the outline, and the teaching idea is clear
	2. The concepts and principles are expounded accurately and highlighted, and the difficulties are handled properly
	3. Grasp the forefront of science, can absorb the latest achievements, to provide relevant information
	4. Do not read the book, and do the theory with practice

Teaching attitude	1. Class and class on time, not absent, do not suspend classes without authorization
	2. Strict requirements for students and patient guidance, answer questions, prepare lessons carefully, timely correct and comment on homework
	3. Be a teacher, rigorous scholarship, teaching, care about students

Teaching method	1. teaching methods are advanced and diversified, such as heuristic, discussion, and case-based teaching methods, to teach students scientific learning methods
	2. Actively and effectively use computer, multimedia and other modern educational technology means to improve the teaching effect
	3. Use Mandarin, and the language is vivid and concise, with a natural teaching attitude
	4. Reasonable arrangement of the course schedule, can make effective use of the class time
	5. The blackboard writing is neat, and the multimedia courseware design is reasonable and beautiful

Teaching efficiency	1. Through teaching, students can master the basic knowledge and skills of the course
	2. Through learning, students' thinking ability has been improved

**Table 2:** Comparison of the classification results of the two binary tree SVM multiple classification algorithms.

Algorithm	Training time (ms)	Testing time (ms)	Precision (%)
The biased binary tree algorithm	23.9	7.1	96.15
The grating method of this paper	24.7	6.5	98.93

## Data Availability

The data used to support the findings of this study are available from the corresponding author upon request.
